RETRACTED

# Exosome-Derived miR-486-5p Regulates Cell Cycle, Proliferation and Metastasis in Lung Adenocarcinoma via Targeting NEK2

**DOI:** 10.3389/fbioe.2020.00259

**Published:** 2020-04-08

**Authors:** Huihui Hu, Hangdi Xu, Fen Lu, Jisong Zhang, Li Xu, Shan Xu, Hanliang Jiang, Qingxin Zeng, Enguo Chen, Zhengfu He

**Affiliations:** ^1^Department of Respiratory and Critical Care Medicine, Sir Run Run Shaw Hospital, School of Medicine, Zhejiang University, Hangzhou, China; ^2^Operation Room, Sir Run Run Shaw Hospital, School of Medicine, Zhejiang University, Hangzhou, China; ^3^Department of Thoracic Surgery, Sir Run Run Shaw Hospital, School of Medicine, Zhejiang University, Hangzhou, China

**Keywords:** miR-486-5p, NEK2, lung adenocarcinoma, proliferation, migration and invasion, cell cycle

## Abstract

**Objective:**

This study aimed to describe the mechanism of exosome-derived miR-486-5p underlying the cell cycle and progression in lung adenocarcinoma (LUAD).

**Methods:**

Bioinformatics methods were applied for identifying the differentially expressed genes (DEGs) in the GEO-LUAD dataset, predicting where the potential target miRNA was expressed and exploring the corresponding downstream target mRNA. qRT-PCR was conducted to detect the levels of the target genes in cancer cells. Thereafter, a series of *in vitro* experiments were performed for cell activities evaluation, including CCK-8, EdU, colony formation assay and transwell. Besides, Western blot was applied to determine the protein levels of the migration and invasion-related factors (NEK2, E-cadherin, N-cadherin, Vimentin, MMP-2, and MMP-9). Dual-luciferase reporter gene assay was employed for validating the targeted relationship between the target genes. Furthermore, nude mouse transplantation tumor experiment was conducted to further validate the role of the target miRNA in tumor development, and immunohistochemistry was used for Ki67 detection and TUNEL was applied for cell apoptosis assay.

**Results:**

miR-486-5p was observed to be enriched in serum exosomes, and seen to be significantly down-regulated in cancer tissues as well as in cancer serum exosomes. It was proven that exosomes could release miR-486-5p, thus regulating LUAD progression and affecting cell cycle. Moreover, NEK2 was identified as a target of miR-486-5p both *in vivo* and *in vitro*. Enrichment analysis revealed that NEK2 was mainly activated in cell cycle and mitosis-related pathways. Meanwhile, NEK2 was found to present significant difference in different TNM stages. Furthermore, rescue experiments indicated that the inhibitory effect of miR-486-5p overexpression on LUAD progression could be abrogated when miR-486-5p and NEK2 were simultaneously up-regulated.

RETRACTED

**Conclusion:**

Exosome-derived miR-486-5p is responsible for cell cycle arrest as well as the inhibition of cell proliferation and metastasis in LUAD via targeting NEK2.

## Introduction

Lung cancer is one of the diseases with the highest incidence and mortality worldwide (Bray et al., 2018). According to the GLOBOCAN 2018 estimates of cancer incidence and mortality produced by the International Agency for Research on Cancer, lung cancer accounts for nearly 11.6% of the total cancer types globally, and it is the leading cause for cancer death with 18.4% of the total (Bray et al., 2018). Non-small cell lung cancer (NSCLC) is the main type of lung cancer accounting for 80–85%. Therein, lung adenocarcinoma (LUAD) is a subtype of NSCLC with the incidence of around 40% in total lung cancer types, and has become increasingly prevalent in the past several decades (An et al., 2017; Wang et al., 2018). Due to the unobvious early symptoms, almost half patients were diagnosed with distant metastasis and the mortality remains high despite the great advance in conventional therapies (Ni et al., 2015). Therefore, it’s necessary to identify LUAD progression-associated genes and mine novel targets for early diagnosis and treatment.

Exosome is a specific subtype of extracellular vesicles (EV) with around 30–100 nm in diameter (Williams et al., 2018; Zhang et al., 2018; Han et al., 2019). Exosomes are present in supernatant of various eukaryotic cells like lymphocytes, epithelial cells, antigen-presenting cells and tumor cells, also in some body fluids, such as blood, amniotic fluid, ascites and urine (Yu et al., 2007; Nilsson et al., 2009; Rupp et al., 2011). Notably, the components and functions of the exosomes depend on the cell types, and exosomes derived from different cells participate in diverse physiological and pathological processes (Yu et al., 2007; Nilsson et al., 2009; Rupp et al., 2011). Recently, many studies have found that tumor cell-derived exosomes can be secreted out of the cells, then migrate away from the primary positions for transferring all types of functional effectors (RNAs, miRNAs, and proteins, etc.) into receptors, thereby resulting in the changes of the tumor microenvironment and consequently affecting the tumor development (Mathivanan et al., 2010; Bai et al., 2019; Monaco et al., 2019). Some serum exosome-derived miRNAs or lncRNAs have been identified to have the potential serving as biomarkers for tumor diagnosis and prognosis. For example, in the serum exosomes of NSCLC patients, lncRNA MALAT-1 is significantly up-regulated and its expression level shows a close correlation with the TNM stages, which demonstrates that exosome-derived MALAT-1 can be used as a non-invasive serum-based tumor biomarker for diagnosis and prognosis of NSCLC (Zhang et al., 2017). Whereas in ovarian cancer, exosome-derived miR-93, miR-145, and miR-200 are all elevated, and miR-145 is confirmed as a potential biomarker for cancer preoperative diagnosis (Kim et al., 2019). But in LUAD, there is an urgent to clarify the molecular mechanism of serum exosomes in tumor development.

miR-486-5p has been proven to act as a tumor suppressor gene in various cancer types. For instance, miR-486-5p suppresses epithelial-mesenchymal transition (EMT) via targeting Snail in prostatic cancer, in turn inhibiting cell metastasis (Zhang et al., 2016). In colorectal cancer, miR-486-5p plays an inhibitory role in tumor cell growth and the formation of lymph vessels through targeting neuropilin-2 (Liu et al., 2016). While in NSCLC, miR-486-5p is regarded as a potential therapeutic target as it can target PIK3RL to attenuate cancer cell growth (Tian et al., 2019). However, the role of exosome-derived miR-486-5p in LUAD remains largely unknown.

RETRACTED

This study sought to investigate the correlation of exosome-derived miR-486-5p with LUAD occurrence and development. Meanwhile, we tried to clarify the relevant underlying mechanism, which helps to explore novel approaches on targeted therapy for LUAD.

## Materials and Methods

### Bioinformatics Analysis

Lung adenocarcinoma microarray GSE36681 was accessed from the GEO database^1^, including 56 pairs of fresh-frozen samples (FF) and 47 pairs of formalin-fixed as well as paraffin-embedded samples (FFPE). “limma” package was utilized to perform differential analysis with the threshold set as | logFC| > 1 and *p*adj < 0.05. The EVmiRNA database was applied to find the positions where the potential differentially expressed miRNA (DEmiRNA) was expressed. Meanwhile, starBase, miRDB and mirDIP three databases were employed for predicting the target genes of the potential DEmiRNA, which were then intersected with the DEmRNAs identified from the TCGA-LUAD^2^ dataset (| logFC| > 2, *p*adj < 0.05). Thereafter, the potential target mRNA was processed for survival analysis combined with the clinical information, followed by GSEA enrichment analysis, so as to investigate the underlying mechanism of the potential serum miRNA and its target mRNA in LUAD.

### Sample Collection

Seurm samples (LUAD: *n* = 76; healthy control: *n* = 76) and tissue samples (tumor: *n* = 76; adjacent normal: *n* = 76) from February 2017 to February 2019 were collected in Sir Run Run Shaw Hospital, College of Medicine, Zhejiang University. Detailed clinical information of all samples was available, and all samples were pathologically diagnosed. Besides, all patients had not received any preoperative radiotherapy or chemotherapy.

RETRACTED

### Cell Culture

Human LUAD cell lines H1650, HCC827, A549, H1975, and PC9, and normal bronchial epithelial cell line BEAS-2B were all purchased from the Research Center of Peking Union Medical College (Beijing, China). All cells were grown in RPMI-1640 mediums (Thermo Fisher Scientific, Waltham, MA, United States) supplemented with 5% fetal bovine serum (FBS; Solarbio, Beijing, China), 100 U/ml of penicillin and 100 μg/ml of streptomycin, and then maintained in 5% CO_2_ at 37°C.

### Cell Transfection

Agomir (miR-486-5p), antagomir (miR-486-5p), oe-NEK2, miR-486-5p mimic and their corresponding negative controls were all procured from Genepharma (Shanghai, China). All cells were seeded in 6-well plates at a density of 3 × 10^5^ cells/well and grown to 50% in confluence for preparation. Meanwhile, 4 ug of target plasmids and 10 ul of Lipofectamin2000 (11668-019, Invitrogen, NewYork, CA, United States) were diluted using 250 ul of serum-free Opti-MEM (51985042, Gibco, Gaitherburg, MD, United States) and sequentially mixed. After 20 min, cells were transfected with the mixture and incubated in 5% CO_2_ at 37°C. The mediums were replaced after 6 h, and cells were collected for follow up analysis after 36–48 h of transfection.

### Exosome Extraction

Human peripheral serum samples were centrifuged twice at 2000rpm for plasmapheresis, and the HIEFF^TM^ Quick exosome isolation kit (41201ES50, Yeasen, Shanghai, China) was used to extract exosomes, following the manufacturer’s instructions. Then, the cell supernatant and isolated exosomes (2:1) were added into the centrifuge tube for incubation overnight at 4°C. On the following day, the mixture was centrifuged at 10000 rpm at 4°C for 1–2 h. The supernatant was removed, whereas the precipitation (exosomes) was collected. Based on the volume ratio of the initial medium and the resuspension (10:1), the precipitation was resuspended in phosphate buffered saline (PBS). Thereafter, 30 μL of the resuspension (exosomes) was placed in an EP tube and then mixed with the Ripa lysis buffer of equal volume and maintained on ice. Microwave methods were employed to lyse the mixture twice and the BCA protein assay kit (Beyotime Biotechnology, Jiangsu, China) was applied for the determination of the protein concentration in exosomes.

### Transmission Electron Microscope (TEM)

Exosomes in suspension were fixed in 0.1 M of calcium carbonite buffer (pH7.4) with 2% glutaraldehyde of equal volume, and then observed under a TEM. The specific procedures were as below: 20 μg of samples were placed on the 300-mesh copper meshes (Agar Scientific Ltd., Stansted, United Kingdom) that were pre-coated with formvar/carbon membranes for adsorption for 2 min. The redundant fluids were absorbed with the filter paper, and 2% phosphotungstic acid was used for counterstaining on the meshes. JEM-1200 exii TEM (JEOL, Tokyo, Japan) was applied to observe the exosomes at 80 kV.

RETRACTED

### Co-culture of Exosomes and LUAD Cells

Cells in logarithmic phase were seeded into 6-well plates that contained 5% FBS (5 × 10^5^ cells/well). Then, 20 μg of exosomes extracted from the transfected A549/H1650 cells and serum was incubated with PKH26 (red; 1:1000) at 37°C for 15 min. Subsequently, PKH26-labeled exosomes were co-cultured with green fluorescent protein (GFP)-labeled LUAD cells in 200 μl of 1% BSC-supplemented PBS, and then maintained at room temperature for 20 min. 4′, 6-diamino-2-phenyl indole (DAPI) was used for staining the nucleoli (blue) of samples, and HelixGen Anti-fade Fluorescence Mounting Medium VECTASHIELD (Vector Labs, CA, United States) was used to block the slides. The Olympus BX61 confocal fluorescence microscope (Zeiss Meta 510, Thornwood, NY, United States) was applied to observe the internalization of exosomes in A549 and H1650 cells.

### qRT-PCR

Total RNA of tissues and cells were extracted using the TRIzol Reagent (Invitrogen), 2 μg of which was then used to be reversely transcribed into cDNA by Superscript II reverse transcriptase (Invitrogen), following the manufacturer’s protocols. The miScript SYBR Green PCR Kit (Qiagen, Hilden, Germany) was applied for the construction of the PCR system, and the Applied Biosystems 7300 Real-Time PCR System (Applied Biosystems, United States) was employed for the examination of miR-486-5p and NEK2 mRNA expression levels. Primers used were synthesized by Sangon Biotech Co., Ltd (Shanghai, Chian) as shown in Table 1. U6 and GAPDH were taken as endogenous controls. 2^–Δ^ ^Δ^ ^Ct^ was used to calculate the relative expression levels of miR-486-5p and NEK2.

**TABLE 1:** Primer Sequences.

**Gene**	**Sequence**
miR-486-5p	F:5′-ACACTCCAGCTGGGTCCTGTACTGAGCTGCCC-3′
	R:5′-CTCAACTGGTGTCGTGGA-3′
NEK2	F:5′- AGATTGGAGCAGAAAGAACAGGAGC-3′
	R:5′-TGCACTTGGACTTAGATGTGAGCTG-3′
U6	F:5′- GTGCAGGGTCCGAGGT-3′
	R:5′- CTCGCTTCGGCAGCACA-3′
GAPDH	F:5′- GGAGCGAGATCCCTCCAAAAT-3′
	R:5′- GGCTGTTGTCATACTTCTCATGG-3′

### CCK-8

The cell counting kit-8 (CCK-8; Beyotime Biotechnology) was used to determine cell proliferation. All cells were planted into 96-well plates (3 × 10^3^ cells/well), and then the CCK-8 reagent was added into each well at 24, 48, 72, and 96 h, respectively. Spectrophotometer was applied to read the OD values at 450 nm at each time point.

RETRACTED

### Colony Formation Assay

Cells were digested with 0.25% trypsin and then suspended by culture mediums. Cells in each group were planted in culture dishes containing 10 ml of culture solution (200 cells/dish). After 3 weeks of routine culture, the mediums were removed when colonies were visible. Thereafter, the colonies were processed for 15 min of fixation with 4% paraformaldehyde and 10 min of staining in 0.1% crystal violet. Being fully stained, the colonies were washed with PBS, and then calculated.

### EdU

Transfected cells were cultured to normal growth in 96-well plates (1 × 10^4^ cells/well). The Cell-Light^TM^ EDU Apollo 488 kit (Ruibio, China) was applied for EdU analysis. Hoechst 33342 was used to stain cells and nucleic acid was identified under a fluorescence microscope. Three fields of each well were randomly chosen for the count of EdU positive cells. The value of the EdU positive cells (red fluorescence)/Hoechest staining cells (blue fluorescence) was calculated for cell proliferation assessment.

### Western Blot

Transfected cells were washed with cold PBS three times for preparation. The whole cell lysate was used to lyse cells for 10 min, and the BCA kit (Thermo, United States) was applied to determine the concentration of the obtained proteins. 30 μg of total proteins were firstly separated by PAGE at 80 V for 35 min followed by 120 V for 45 min, and then transferred onto the PVDF membranes (Amersham, United States). After being blocked in 5% skim milk at room temperature for 1 h, the membranes were incubated together with primary antibodies overnight at 4°C, sequentially cultured with horseradish peroxidase (HRP)-labeled secondary antibody goat anti-rabbit IgG H&L (ab6721, 1:3000, abcam, Cambridge, United Kingdom) at room temperature for 1 h. PBST (PBS buffer containing 0.1% Tween-20) was used to wash the membranes after each reaction. The protein bands were visualized using an optical luminometer (GE, United States), and analyzed by the Image Pro Plus 6.0 (Media Cybernetics, United States) software.

Primary antibodies included CD63 (ab68418, 1 μg/ml, abcam, Cambridge, United Kingdom), CD81 (ab155760, 1:2000, abcam, Cambridge, United Kingdom), Alix (ab76608, 1 μg/ml, abcam, Cambridge, United Kingdom), NEK2 (ab115731, 1:1000, abcam, Cambridge, United Kingdom), N-cadherin (ab76057, 1:1000, abcam, Cambridge, United Kingdom), E-cadherin (ab15148, 1:500, abcam, Cambridge, United Kingdom), Vimentin (ab137321, 1:2000, abcam, Cambridge, United Kingdom), MMP-2 (ab37150, 1 μg/ml, abcam, Cambridge, United Kingdom), MMP-9 (ab38898, 1:1000, abcam, Cambridge, United Kingdom) and GADPH (ab9485, 1:2500, abcam, Cambridge, United Kingdom). All antibodies were rabbit polyclonal antibodies.

RETRACTED

### Transwell

#### Migration Assay

Cells in logarithmic phase were harvested in serum-free mediums for 24 h. On the following day, cells were digested, centrifuged and resuspended to a final concentration of 2 × 10^5^ cells/mL. 0.2 ml of cell suspension was put into the Transwell inserts, and 700 μL of pre-cooled DMEM containing 10% FBS was placed under the inserts. After 24 h of incubation in 5% CO_2_ at 37°C, cells still in the inserts were wiped off using a cotton swab, whereas cells migrated out of the inserts were fixed by methanol for 30 min and stained in 0.1% crystal violet for 20 min. Cells were observed under an inverted microscope and photographed, then five fields were chosen at random for cell count.

#### Invasion Assay

24-well Transwell inserts (8 μm in aperture, BD Biosciences) were applied for cell invasion assay. Around 2 × 10^4^ cells were placed into the Matrigel matrix-coated (Corning, NY, United States) upper chambers, and DMEM supplemented with 10% FBS was added into the lower chambers. The follow-up specific procedures were similar as the migration assay above.

### Flow Cytometry

#### Cell Apoptosis Assay

Cells were cultured in 6-well plates and then collected for transfection when the density reached 2 × 10^4^ cells/well. After 48 h, cells were harvested after being digested by EDTA-free trypsin, and then resuspended in PBS at 4°C. Thereafter, the cell suspension was centrifuged at 1000rpm at 4°C, and resuspended again in 1 × binding buffer. Annexin V-FITC apoptosis assay kit (Biovision, K101) was applied to detect cell apoptosis within 15 min in dark. Flow cytometry (BD Biosciences) was employed to calculate the apoptotic rate.

#### Cell Cycle Assay

Transfected cells were grown in dishes (6 cm; 2 × 10^5^ cells/dish) until 80% in confluence. Then the cells were digested by trypsin, washed with cold PBS and collected. After being fixed by 75% ethanol, cells were treated with RNase A (Sigma-Aldrich) and stained in 500 μL PI (Sigma-Aldrich). Flow cytometry (Beckman-Coulter) was utilized to analyze the cell distribution in each phase, and the cells in G0/G1, S and G2/M phase in each group were count and compared.

### Dual-Luciferase Reporter Gene Assay

Amplified mutant and wild type NEK2 3′UTR (NEK2 3′UTR-MUT and NEK2 3′UTR-WT) were cloned into luciferase pmirGLO vectors (Promega, WI, United States) for building of NEK2-WT and NEK2-MUT vectors. Renilla luciferase expression vector pRL-TK (TaKaRa, Dalian, China) was used as the internal reference. Each plasmid was co-transfected with either NEK2-WT or NEK2-MUT into HEK-293T cells, and the luciferase activity was determined by Dual-Luciferase Reporter Assay System (Promega, Madison, WI, United States).

RETRACTED

### Nude Mouse Transplantation Tumor Experiment

Totally 24 BALB/c female nude mice (3–4 weeks, 15 ± 2 g in weight) were selected and housed in a constant environment (25–27°C, 45–50% humidity). All mice were divided equally at random with 12 mice in each group. All procedures were conformed to the ethics convention released by the International Council for Laboratory Animal Science, and complied with the related national regulations. oe-NC or oe-NEK2-transfected cells (20 μL, 1 × 10^7^ cells/mL) were subcutaneously injected into the nude mice, and tumor growth was observed every 6 days and the images were captured. Survival curve based on the tumor volume was plotted and formulated as (a × b^2^)/2 (*a* = the longest diameter, *b* = the shortest diameter). After 30 days, the nude mice were executed and the transplanted tumors were isolated for weight measurement. Tissues from the transplanted tumors were extracted for subsequent qRT-PCR and immunohistochemistry experiments.

### Immunohistochemistry

Sections of transplanted tumors were obtained for immunohistochemistry. Samples were firstly treated with 3% hydrogen peroxide for 10 min, and then rinsed with distilled water and PBS. 0.01 M sodium citrate buffer (pH6.0) was added into the samples for antigen retrieval for 15 min, and then the samples were washed in PBS. After being blocked in normal goat serum for 30 min, the samples were incubated with primary antibodies overnight at 4°C, followed by secondary antibody at room temperature for 60 min. Samples with PBS were taken as the negative control. DAB was used to stain the samples (3–10 min) and hematoxylin was added for counterstaining. 0.5% acid alcohol was used for color separation. After neutralization using alkali for 30–60 s, the samples were rinsed in running water for 15 min, washed in distilled water twice, then dehydrated, blocked and observed under a microscope. Primary antibodies included NEK2 (ab115731, 2.5 μg/ml, abcam, Cambridge, United Kingdom) and Ki67 (ab15580, 1 μg/ml, abcam, Cambridge, United Kingdom). The secondary antibody was horseradish peroxidase (HRP)-labeled goat anti-rabbit IgG H&L (ab6721, 1:3000, abcam, Cambridge, United Kingdom). All antibodies were rabbit polyclonal antibodies.

### Statistical Analysis

All data were processed through the SPSS 21.0 software (SPSS, Inc., Chicago, IL, United States). Mean ± standard deviation was used to express the measurement data, and Student’s *t* test as well as the one-way analysis of variance (ANOVA) was applied for the assessment of group comparisons. Data at different time points were analyzed in repeated measures ANOVA and validated in tukey’s test. Kaplan-Meier and log-rank analyses were performed for the overall survival assessment. Count data were analyzed by chi-square test. Each result was representative of at least three independent experiments. *P* < 0.05 was considered statistically significant, while *p* < 0.01 was regarded extremely statistically significant.

RETRACTED

## Results

### miR-486-5p Is Mainly Observed in Serum Exosomes and Is Poorly Expressed in LUAD

According to the differential analysis, a total of 7 DEmiRNAs were identified from FF samples in GSE36681, and 2 DEmiRNAs from FFPE samples (Figure 1A). Among them, miR-486-5p was found to be significantly down-regulated in both the two types of samples. Besides, miR-486-5p was seen to be enriched in serum exosomes using the EVmiRNA database (Figure 1B). Published literatures have suggested that serum exosomes are responsible for the tumorigenesis and development of NSCLC (Grimolizzi et al., 2017; Kanaoka et al., 2018). Meanwhile, serum-derived miR-486 has been reported to have the potential serving as a biomarker in cervical cancer diagnosis (Li et al., 2018). In addition, we found that miR-486-5p exhibited the most remarkable difference in LUAD tissues and adjacent normal tissues relative to other types of tumors in TCGA database (Figure 1C).

**FIGURE 1:** miR-486-5p is mainly observed in serum exosomes and poorly expressed in LUAD. In all, **(A, left)** 7 DEmiRNAs were identified from FF samples in GSE36681, and **(A, right)** 2 DEmiRNAs from FFPE samples. The **(A)** expression difference of these DEmiRNAs in tumor tissues and normal cases were plotted in heatmaps. EVmiRNA database was used to detect the **(B)** expression levels of miR-486-5p in exosomes derived from various tissues, finding that miR-486-5p was mainly expressed in serum exosomes. Besides, **(C)** miR-486-5p expression in diverse tumor tissues included in TCGA database was accessed. Exosomes in LUAD serum and normal serum were observed under a **(D)** TEM, and **(E)** western blot was performed to determine the levels of exosome protein markers CD63, CD81, and Alix. qRT-PCR was conducted to test miR-486-5p in **(F)** LUAD serum, **(G)** tumor tissues and the normal counterparts, also in **(H)** LUAD cell lines H1650, HCC827, A549, H1975, PC9 and normal bronchial epithelial cell BEAS-2B. (*P < 0.05, **P < 0.01).

Exosomes of normal people and LUAD patients were extracted and observed under a TEM as shown in Figure 1D. Western blot was performed for detecting the levels of exosome protein markers CD63, CD81 and Alix, indicating that exosomes were successfully extracted (Figure 1E). Then, qRT-PCR was conducted and found that miR-486-5p was greatly down-regulated in LUAD serum exosomes relative to that in normal counterparts (Figure 1F). As well, the expression of miR-486-5p in tumor tissues was significantly lower than that in adjacent normal tissues (Figure 1G), which was consistent with the bioinformatics analysis result. Notably, miR-486-5p showed a similar expression trend in LUAD cells relative to the normal bronchial epithelial cell BEAS-2B (*p* < 0.05), and the lowest expression was present in A549 and H1650 cells (*p* < 0.01) (Figure 1H). Thus, A549 and H1650 cells were selected for subsequent experiments, and A549 was used for nude mouse transplantation tumor model experiment.

RETRACTED

### Serum Exosomes Suppress LUAD Progression

To explore the role of serum exosomes in LUAD cell proliferation, migration, invasion and cell cycle, A549 and H1650 cells were divided into the NC group (PBS) and exosome group (normal people). As observed by the confocal microscope, exosomes were internalized by LUAD cells and distributed around the nuclei (Figure 2A). Then, cell proliferation in each group was assayed by a series of experiments. EdU assay revealed that the EdU positive rate was remarkably decreased in exosome group, suggesting the inhibition of DNA replication (Figure 2B). Meanwhile, CCK-8 showed that the cell proliferation rate in exosome group was significantly lower than that in the NC group (Figure 2C), and colony formation assay showed that the number of colony was significantly reduced in the exosome group relative to the NC group (Figure 2D). Thereafter, flow cytometry was carried out to determine cell apoptosis and cell cycle. As shown in Figure 2E, cell apoptotic rate was greatly increased in the exosome group relative to the NC group. As well, cells in the exosome group were mainly accumulated in G0/G1 phase, whereas there was fewer cells in the S phase (Figure 2F). Moreover, Transwell assay was performed and found that cells in the exosome group had poorer migration and invasion abilities in comparison with the NC group (Figure 2G). In addition, to further investigate the effect of serum exosomes on tumor metastasis, the protein levels of EMT-related markers and matrix hydrolase were detected through western blot. As plotted in Figure 2H, in the exosome group, N-cadherin and Vimentin were decreased, whereas E-cadherin was increased (*p* < 0.05), which indicated the impeding of EMT process. Meanwhile, migration-related proteins MMP2 and MMP9 were also observed to be greatly reduced (*p* < 0.05). Furthermore, the expression of miR-486-5p was seen to be elevated in the exosome group via qRT-PCR (Figure 2I). Taken together, the above findings demonstrated that serum exosomes were responsible for the suppression of cell proliferation, migration and invasion, as well as for the promotion of cell apoptosis and cell cycle arrest in LUAD in an internalization manner.

RETRACTED

**FIGURE 2:** Serum exosomes suppress LUAD progression. As observed by a **(A)** confocal microscope (×400), exosomes were internalized by LUAD cells and distributed around the nuclei. PKH26-labeled exosomes are red, GFP-labeled A549/H1650 are green. Exosomes were used to co-culture with cells, and then the cells were harvested for EdU (**B:** DNA replication, 200×), CCK-8 (**C:** cell proliferation), colony formation assay (**D:** colony forming ability), flow cytometry (**E:** cell apoptosis; **F:** cell cycle), and transwell (**G:** migration and invasion). Western blot was carried out to determine the **(H)** EMT-related proteins E- cadherin, N-cadherin, Vimentin, MMP-2 and MMP-9, and the **(I)** miR-486-5p in exosome co-cultured cells were also detected by qRT-PCR. (^#^,*p < 0.05, **p < 0.01).

### miR-486-5p Inhibits Cell Proliferation and Metastasis in LUAD as Well as Makes Cell Cycle Arrest

As above mentioned, miR-486-5p was elevated in cells co-cultured with cancer serum exosomes (Figure 2I). Hence, we reasoned that exosomes might function on tumor development via releasing miR-486-5p. miR-486-5p agomir, miR-486-5p antagomir and their negative controls were transfected into cells for construction of miR-286-5p overexpression and silencing. EdU, CCK-8 and colony formation assay were all suggested that cells in the miR-486-5p agomir group had the poorest proliferation ability, but the strongest ability in the miR-486-5p antagomir group (Figures 3A–C). Besides, flow cytometry revealed that miR-486-5p overexpression significantly increased cell apoptotic rate, and opposite result was observed when miR-486-5p was silenced (Figure 3E). Meanwhile, cell cycle was test as shown in Figure 3F, finding that cell cycle was arrested in G0/G1 phase in the miR-486-5p agomir group. Reversely, cell cycle was accelerated accompanied by the increase of the cell proliferation rate in the miR-486-5p antagomir group, as evidenced by the remarkably decreased cell proportion in G0/G1 phase. Furthermore, cell migration and invasion were assayed, finding the greatly reduced migrated and invasive cells in the miR-486-5p agomir group, but remarkably increased cells in the miR-486-5p antagomir group (Figure 3D). To make the results more receivable, EMT and metastasis-associated proteins N-cadherin, Vimentin, MMP2 and MMP9 were detected and all showed significantly down-regulated levels in the miR-486-5p agomir group, whereas opposite result was shown in the miR-486-5p antagomir group (Figure 3G). Collectively, the results shed light on the inhibitory role of miR-486-5p in cell proliferation, migration and invasion, but a promotive role in cell apoptosis.

RETRACTED

**FIGURE 3:** miR-486-5p inhibits cell proliferation, metastasis and induces cell apoptosis in LUAD, and makes cell cycle arrest. miR-486-5p agomir, miR-486-5p antagomir and their negative controls were transfected into H1650 and A549 cell lines, and then cells were collected for the detection of cell proliferation by **(A)** EdU, **(B)** CCK-8 and **(C)** colony formation assay, and for the examination of panel **(D)** cell migration and invasion by transwell, also for assessment of panel **(E)** cell apoptosis as well as **(F)** cell cycle by flow cytometry. Western blot was carried to determine the **(G)** EMT-related proteins E- cadherin, N-cadherin, Vimentin, MMP-2 and MMP-9. (*p < 0.05, **p < 0.01).

### miR-486-5p Targeted Down-Regulates NEK2 in LUAD

In all, 1975 up-regulated DEmRNAs and 528 down-regulated DEmRNAs were identified in the TCGA-LUAD dataset. starBase, miRDB and mirDIP three databases were used to predict the target mRNAs of miR-486-5p. Venn diagram was plotted and eventually four DEmRNAs bearing targeted binding sites with miR-486-5p were obtained (Figure 4A). Correlation analysis revealed that there was an extremely significant negative correlation between miR-486-5p and NEK2, as suggested by the highest pearson correlation coefficient (Figure 4B). Meanwhile, miR-486-5p and NEK2 were also seen to be reversely correlated in the expression level (Figure 4C). When miR-486-5p was overexpressed, NEK2 was detected to be greatly suppressed (Figure 4I). To further validate the targeted relationship between the two factors, dual-luciferase assay was performed and found that the luciferase activity was remarkably attenuated in cells with NEK2-WT after miR-486-5p was overexpressed, while there was no difference observed in cells with NEK2-MUT (Figure 4J). In sum, miR-486-5p could targeted regulate NEK2.

**FIGURE 4:** miR-486-5p targeted down-regulates NEK2 in LUAD. **(A)** Venn diagram was plotted to find the target mRNAs, and eventually 4 mRNAs were obtained, among which NEK2 showed the highest **(B)** pearson correlation coefficient with miR-486-5p (red means positive correlation, blue means negative correlation). Besides, **(C)** correlation analysis revealed that there was a negative correlation between miR-486-5p and NEK2. Thereafter, to explore the role of NEK2 in LUAD, NEK2 was test in **(D)** LUAD tissue samples and adjacent normal tissues as plotted in a Boxplot. **(E)** Survival analysis was performed on NEK2 in the TCGA-LUAD dataset, finding that NEK2 high expression predicted poor prognosis, with red representing high expression and blue representing low expression. **(F)** GSEA enrichment analysis suggested that NEK2 was mainly activated in cell cycle and mitosis-related pathways. Then, NEK2 expression was measured in **(G)** patients with different TNM stages and in **(H)** BEAS-2B, HCC827 and A549 cells by qRT-PCR. To further investigate the relationship between miR-486-5p and NEK2, NEK2 was detected **(I)** in H1650 and A549 cells in protein level by western blot. In addition, **(J)** starBase database was used to predict the binding sites of miR-486-5p on NEK2 and dual-luciferase assay was conducted to further validate such targeted relationship. (*p < 0.05, **p < 0.01).

RETRACTED

Subsequently, the role of NEK2 in LUAD was further investigated. qRT-PCR showed that NEK2 was profoundly up-regulated in both LUAD tissue samples and cells relative to the normal counterparts (Figures 4D,H). As well, there was a significant difference in NEK2 level in different TNM stages, presenting as a positive correlation between NEK2 level and the staging grade (Figure 4G). In addition, Kaplan-Meier analysis revealed that NEK2 high expression predicted the poor survival (Figure 4E). And GSEA enrichment analysis suggested that NEK2 was mainly enriched in cell cycle and mitosis-related pathways (Figure 4F). In general, NEK2 had the potential serving as an oncogene in LUAD.

### miR-486-5p Functions in LUAD Progression via Targeting NEK2

Rescue experiments were conducted to further explore the underlying mechanism of miR-486-5p/NEK2 in LUAD proliferation and metastasis. Cells were classified into three groups: miR-486-5p agomir + oe-NEK2, miR-486-5p agomir + oe-NC and NC agomir + oe-NC. Firstly, qRT-PCR was performed to detect the transfection efficiency and found that NEK2 was significantly reduced in the miR-486-5p agomir + oe-NC group relative to the NC agomir + oe-NC group, but remarkably increased in the miR-486-5p agomir + oe-NEK2 group as compared to the miR-486-5p agomir + oe-NC group (Supplementary Figure S1). CCK-8 and colony formation assay were performed, finding that cells in the miR-486-5p agomir + oe-NEK2 group were determined to have much higher proliferation rate as well as colony formation rate than that in the miR-486-5p agomir + oe-NC group (Figures 5A,B). In addition, flow cytometry showed that miR-486-5p overexpression could induce apoptosis in LUAD, and such promotive effect could be reversed when NEK2 was concurrently overexpressed (Figure 5C). Similarly, the inhibitory effect of miR-486-5p overexpression on cell migration and invasion could also be abrogated under the condition of NEK2 overexpression (Figure 5D). Moreover, we test the levels of migration-associated proteins, and found that only E-cadherin was reduced in the miR-486-5p agomir + oe-NEK2 group in comparison with the miR-486-5p agomir + oe-NC group, while N-cadherin, Vimentin, MMP2 and MMP were all elevated (Figure 5E). In all, the effects of miR-486-5p overexpression on cell proliferation, migration, invasion and apoptosis could be abolished in a NEK2 overexpression manner.

RETRACTED

**FIGURE 5:** miR-486-5p functions on LUAD progression and affects cell cycle via targeting NEK2. miR-486-5p agomir + oe-NEK2, miR-486-5p agomir + oe-NC and NC agomir + oe-NC were transfected into H1650 and A549 cells, and then cells were harvested for the determination of cell proliferation by **(A)** CCK-8 and **(B)** colony formation assay, for the detection of panel **(C)** cell apoptosis and **(F)** cell cycle by flow cytometry, and for the test of panel **(D)** migration and invasion by transwell. Also, **(E)** EMT-related proteins E- cadherin, N-cadherin, Vimentin, MMP-2 and MMP-9 were detected by western blot. (#,*p < 0.05, **p < 0.01).

As previously analyzed, NEK2 were predominantly activated in cell cycle and mitosis-related pathways. Thus, to determine the role of miR-486-5p/NEK2 in cell cycle in LUAD, flow cytometry was carried out on these three groups. As shown in Figure 5F, cells in the miR-486-5p agomir + oe-NC group were greatly accumulated in G0/G1 phase, suggesting that the overexpression of miR-486-5p could arrest cell cycle into S phase, thereby suppressing cell proliferation. Yet such effect was attenuated when miR-486-5p and NEK2 were simultaneously overexpression processed. Taken together, the findings elucidated that miR-486-5p could regulate cell cycle in LUAD via targeting NEK2.

### miR-486-5p Overexpression Plays an Inhibitory Role in Tumor Formation in LUAD *in vivo*

Nude mouse models were constructed to seek the effect of miR-486-5p on tumor development *in vivo*. A549 cells were divided into miR-486-5p agomir group and NC agomir group. After that tumor transplantation was carried out, tumor weight and volume were monitored every 6 days. 30 days later, both weight and volume in the miR-486-5p agomir group were significantly smaller than those in NC controls (Figure 6A), suggesting that the tumor growth was inhibited. Meanwhile, miR-486-5p was detected to be successfully overexpressed in the miR-486-5p agomir group by qRT-PCR (Figure 6B). Thereafter, NEK2 level was examined and observed to be remarkably decreased both in mRNA and protein levels in the miR-486-5p agomir group (Figures 6C,D). Besides, same result could be obtained by immunohistochemistry, and the Ki67 positive rate in the miR-486-5p agomir group was much lower relative to the NC agomir group (Figures 6E,F). In short, the overexpression of miR-486-5p was capable of down-regulating NEK2 in transplanted tumors, thus contributing to the inhibition of cell proliferation.

RETRACTED

**FIGURE 6:** miR-486-5p overexpression plays an inhibitory role in tumor formation in LUAD *in vivo.* miR-486-5p agomir-transfected A549 cells were planted into nude mice, and **(A)** tumor weight and volume were monitored every 6 days. After 30 days, the tumors were isolated. **(B)** qRT-PCR was performed to detect the transfection efficiency. Then, NEK2 was measured by **(C)** qRT-PCR and **(D)** western blot, finding that NEK2 was significantly down-regulated both in mRNA and protein levels, which was further validated by immunohistochemistry (**E:** NEK2 expression; **F:** Ki67 positive rate). The **(D)** EMT-related proteins E-cadherin, N-cadherin, Vimentin, MMP-2 and MMP-9 were sequentially test for further exploring the effect of miR-486-5p overexpression on cell metastasis. (*p < 0.05).

Migration-related proteins were detected for validating the role of miR-486-5p overexpression in tumor metastasis *in vivo*, and the result was plotted in Figure 6D. Consistent with the *in vitro* experiment, E-cadherin showed a high expression when miR-486-5p was overexpressed, whereas N-cadherin, Vimentin, MMP2 and MMP9 exhibited a low expression. This result demonstrated that miR-486-5p overexpression could function on cell metastasis in LUAD via suppressing EMT process.

## Discussion

Lung adenocarcinoma is a subtype of NSCLC with great advances that have been made in diagnosis and treatment in recent years, yet the clinical prognosis and the overall survival were still poor (Siegel et al., 2019). Hence, it’s a necessity to further investigate the underlying mechanism in LUAD progression, and seek for novel biomarkers for targeted diagnosis and therapy. Recently, exosomes have been deeply researched, and increasing evidence has suggested that exosomes play important roles in cell communication, tumorigenesis, tumor metastasis and microenvironment (Feng et al., 2019; Samuel and Gabrielsson, 2019; Yu et al., 2019). Notably, exosomes can function on tumor progression through releasing miRNAs to receptors in an internalization manner, and exosomes derived from diverse cells work different (De Feo et al., 2019; Kulkarni et al., 2019; Liu et al., 2019). For example, in colorectal cancer, mesenchymal stem cell-derived exosomes are responsible for the suppression of cell proliferation, migration and invasion via the miR-16-5p/ITGA2 axis (Xu et al., 2019). While in NSCLC, A549-drug resistance-derived exosomes can promote the parent cell proliferation, migration, invasion and enhance the drug resistance of patients to gemcitabine via the miR-222-3p/SOCS3 axis (Wei et al., 2017). In our study, we found that miR-486-5p was mainly enriched in serum exosomes through bioinformatics methods. Besides, miR-486-5p was seen to be remarkably decreased in LUAD serum exosomes and tumor tissues relative to the normal counterparts. Our findings shed light on that exosome-derived miR-486-5p in serum can be utilized as a potential biomarker for LUAD diagnosis, which highlights the importance of the investigation on the molecular mechanism in LUAD progression.

RETRACTED

In addition, we further explored the effects of miR-486-5p on LUAD cell proliferation and metastasis. Prior studies have proven that miR-486-5p plays a regulatory role in the development and drug resistance of various cancer types. For instance, miR-486-5p can regulate the production and potentiate the growth of normal red blood cells, and it can mediate the drug response of chronic myeloid leukemia progenitor cells (Wang et al., 2015). Whereas in renal cell carcinoma, miR-486-5p is decreased by interacted with the CCL2 (C-C motif chemokine ligand 2) of tumor-related macrophages, and miR-486-5p restoration is capable of inhibiting cell proliferation and inducing cell apoptosis (He et al., 2019). However, the role of miR-486-5p in LUAD remains poorly studied. In the present study, we discovered that exosomes could pass miR-486-5p to LUAD cells, thus achieving the purpose of suppressing cell proliferation, migration, invasion and promoting cell apoptosis. In addition, *in vivo* experiments confirmed that miR-486-5p overexpression played an inhibitory role in tumor formation as well as metastasis. The results revealed that miR-486-5p had the potential acting as a tumor suppressor gene in LUAD.

Multiple studies have indicated that miRNAs act as key mediators in tumor signal transduction pathways, with the behaviors of degrading or inhibiting their target mRNAs (He et al., 2015; Zhou et al., 2016). Dual-luciferase reporter gene assay showed that miR-486-5p targeted NEK2 and down-regulated NEK2 expression both *in vivo* and *in vitro*. Moreover, we performed qRT-PCR and found that NEK2 was significantly elevated in tumor tissues. Matched clinical information was also obtained and analyzed, finding that NEK2 was remarkably correlated with TNM stages and prognosis, as indicated by that NEK2 expression was increased with the higher grade of TNM staging and NEK2 high expression was always in concomitant with poor prognosis. NEK2 has been reported to function as an oncogene in diverse cancers, and it exhibits an intimate correlation with the drug resistance of tumors. In hepatocellular carcinoma (HCC), for example, NEK2 activates the transcription of downstream target genes through stabilizing β-catenin and promoting its translocation to the nucleus, consequently enhancing the sorafenib resistance in HCC cells (Deng et al., 2019). Fan et al. (2019) reported that NEK2 potentiated the malignant proliferation of gastric cancer cells via the ERK/MAPK axis. In our study, we validated that miR-486-5p targeted NEK2 to regulate LUAD progression, and simultaneous overexpression of miR-486-5p and NEK2 could rescue the inhibitory effect of miR-486-5p on cancer cell activities.

RETRACTED

KEGG and GO enrichment analyses were conducted and revealed that NEK2 was mainly enriched in cell cycle and mitosis-related pathways. Many studies have suggested that NEK2 is a kinase implicated in regulating the S/G2 phase in cell cycle (Pfleger and Kirschner, 2000; Weber and Mlodzik, 2017). Notably, NEK2 is involved in the separation of centrosomes. Besides, there is no NEK2 expression observed in G1 phase, but increased expression in S phase, and in G2 phase the expression is elevated to peak (Fry et al., 1998, 2012; Hames et al., 2001). In addition, NEK2 is responsible for the suppression of primary cilia formation (Spalluto et al., 2012; Kim et al., 2015). In this study, we discovered that miR-486-5p overexpression induced cell cycle arrest in G0/G1 phase via targeting NEK2, leading to the inhibition of cell proliferation. Meanwhile, the cell proportion in S and G2 phases were increased when NEK2 was concurrently overexpressed, as well, cell proliferation ability was recovered and the promotive effect of miR-486-5p overexpression on cell apoptosis was in turn reversed.

## Conclusion

Our study found the relative lower expression of miR-486-5p in LUAD tissues and serum exosomes, and confirmed that exosomes exerted their role sin cell proliferation, migration, invasion and apoptosis in LUAD in a miR-486-5p manner. Moreover, NEK2 was identified as a target of miR-486-5p and found to be activated in cell cycle-related pathways. miR-486-5p played a key role in regulating LUAD development via targeting NEK2, which provides a novel target for future LUAD diagnosis and treatment.

## Data Availability Statement

All datasets generated for this study are included in the article/Supplementary Material.

## Ethics Statement

This study was conducted in accordance with the Helsinki Declaration II and was approved by the Institutional Review Boards of Sir Run Run Shaw Hospital, College of Medicine, Zhejiang University.

## Author Contributions

HH, HX, and FL designed the study. JZ and LX conducted the literature search. SX and HJ wrote the manuscript. QZ performed the data analysis. EC, HH, and ZH revised the manuscript. All authors gave the final approval of the version to be submitted.

RETRACTED

## Conflict of Interest

The authors declare that the research was conducted in the absence of any commercial or financial relationships that could be construed as a potential conflict of interest.

## Footnotes

1 https://www.ncbi.nlm.nih.gov/geo/

2 https://portal.gdc.cancer.gov/

## Supplementary Material

FIGURE S1 Transfection of NEK2 rescued the miR-486-5p-induced downregulation of NEK2.
